The article "By up-regulating μ- and δ-opioid receptors, neuron-restrictive silencer factor knockdown promotes neurological recovery after ischemia" was retracted in 2025. Reasons: plagiarized images; overlap with other authors' work.

# By up-regulating μ- and δ-opioid receptors, neuron-restrictive silencer factor knockdown promotes neurological recovery after ischemia

**DOI:** 10.18632/oncotarget.18195

**Published:** 2017-05-23

**Authors:** Hui-Min Liang, Li-Jiao Geng, Xiao-Yan Shi, Chao-Gang Zhang, Shu-Yan Wang, Guang-Ming Zhang

**Affiliations:** ^1^ Department of Neurology, Huaihe Hospital of Henan University, Kaifeng 475000, China; ^2^ Institute of Traditional Chinese Medicine, Henan University, Kaifeng 475000, China; ^3^ Department of Anesthesiology, Tongren Hospital, Shanghai Jiao Tong University School of Medicine, Shanghai 200336, China

**Keywords:** neuron-restrictive silencer factor, cerebral ischemia, μ- and δ-opioid receptors, proliferation, apoptosis

## Abstract

We investigated the effects of neuron-restrictive silencer factor (NRSF) on proliferation of endogenous nerve stem cells (NSCs) and on μ- and δ-opioid receptor (MOR/DOR) expression in rats after cerebral ischemia. Among 100 rats subjected to cerebral ischemia, 20 rats were transfected with NRSF shRNA, and the remaining 80 were randomly assigned to normal, sham, model, and negative control (NC) groups. On days 7, 14, and 28 after ischemia and reperfusion, neurological function scores were assigned and a step-down passive avoidance test was conducted. Nerve function scores, step-down reaction periods, error times and apoptosis rates, as well as levels of B-cell CLL/lymphoma 2 (Bcl-2), BCL2-associated X protein (Bax), and NRSF expression were lower in the NRSF shRNA group than in the model and NC groups. By contrast, step-down latency, numbers of bromodeoxyuridine-positive cells, MOR/DOR expression, and phosphorylation of extracellular signal regulated protein kinase (ERK) and cAMP response element binding protein (CREB) were higher in the NRSF shRNA group than in the model and NC groups. These results suggest that by up-regulating MOR/DOR expression, NRSF knockdown accelerates recovery of neurological function after cerebral ischemia, at least in part by promoting NSC proliferation and inhibiting apoptosis.

## INTRODUCTION

Cerebral ischemic injuries (ischemic strokes) are one of the most common cerebral vascular diseases and have a morbidity rate second only to malignant tumors [1]. Ischemic strokes are large-scale events that are responsible for around 80% of all stroke cases and result in irreversible damage, including neuronal injury and death [2]. Many factors such as inflammation, apoptosis, oxidative stress, intracellular calcium overload, and excitatory amino acid toxicity, are involved in the pathological effects of ischemic strokes [3]. Currently, the main treatments for cerebral ischemia injury include thrombolytic therapy and a variety of protective agents that aim to prevent brain cell apoptosis and enhance neuro-protective processes [4]. Apoptosis and inflammation are the two largest contributors to cerebral ischemic injury, and many studies have focused on related molecular therapies that inhibit apoptosis and attenuate inflammation [5–7].

Neuron-restrictive silencer factor (NRSF), also called RE1-silencing transcription factor (REST), is a member of the Kruppel-type zinc-finger family and a negative regulator of neuronal gene transcription [8]. NRSF, which is highly expressed outside of the nervous system, is absent from neuronal cells and silences the expression of the neuron-specific genes superior cervical ganglion 10 (SCG10) and type II voltage-dependent sodium channel gene, indicating that it is able to bind 24-bp cis-elements [9]. NRSF acts as a crucial determinant of progenitor cell fate by inhibiting the transcription of neuron-specific genes [10].

The μ- and δ-opioid receptors (MOR/DOR) are two of the three class A G protein-coupled opioid receptors [11]. Activation of these opioid receptors inhibits adenylyl cyclase and voltage-gated Ca^2+^ channels. This in turn increases mitogen-activated protein kinase (MAPK) phosphorylation [12] and stimulates the transcription of genes that regulate cellular differentiation, proliferation, and survival [13]. Choi *et al* found that the type 2 cannabinoid receptor (CB2R), which upregulates the AMPK/CREB pathway, is a potential therapeutic target for cerebral ischemia injury [14]. Additionally, previous studies have demonstrated that MOR/DOR activation increases tolerance against cerebral ischemia and reduces ischemia injury [15, 16]. NRSF also post-transcriptionally represses the *MOR* gene in neuronal cells [17]. We therefore used a cerebral ischemia rat model to examine whether NRSF affects the proliferation of endogenous nerve stem cells (NSCs) by regulating MOR/DORs.

## RESULTS

### CBF in the rat cortex after ischemia

During ischemia, local cerebral blood flow (CBF) in the parietal cortex sharply declined to less than 30% of the pre-ischemia level. CBF remained at this reduced level for the 1 hr duration of ischemia and only partially recovered during reperfusion. This indicates that the ischemia model was successful (Figure 1).

**Figure 1:** Changes in local CBF in the parietal cortex of model group rats CBF: cerebral blood flow.

### Expression of NRSF mRNA and protein after NRSF knockdown

qRT-PCR demonstrated that NRSF mRNA expression was lower in the NRSF shRNA group and higher in the model group than in the normal and sham groups (*P* < 0.05, Figure 2A). Western blots demonstrated that NRSF protein levels were lower in the NRSF shRNA group and higher in the model group than in the normal and sham groups (*P* < 0.05, Figure 2B).

**Figure 2:** (**A**) NRSF mRNA expression in each group. (**B**) protein expressions of NRSF and β-actin in each group detected by western blot. (**C**) NRSF protein expression in each group. ^*^P < 0.05 compared to the normal group; ^#^*P* < 0.05 compared to the model group; NC, negative control; NRSF, neuron-restrictive silencer factor.

### NRSF knockdown promotes recovery of nerve function scores after ischemia

The results of neurological function scoring for all groups are shown in Table 1. The rats in the normal and sham groups displayed no neurologic deficits with scores of 0. The rats in the model, NC, and NRSF shRNA groups presented different degrees of neurologic deficits and all had scores higher than 0. As reperfusion continued, symptoms of neurologic deficits began to disappear; scores were lower in both the model and NC groups on the 28th day compared to the previous time point (both *P* < 0.05). The only decreases in scores compared to the previous time point among all of the groups occurred in the NRSF shRNA group on the 14th and 28th days (*P* < 0.05). Scores did not differ between the model and NC groups at any of the time points, and scores for the NRSF shRNA group were lower than those of both the model and NC groups at all time points (all *P* < 0.05). These results demonstrated that NRSF knockdown accelerated the recovery of neurological function.

**Table 1:** Comparison of the nerve function scores of the rats after ischemia among the normal, sham, model, NC and NRSF shRNA groups ($\bar{\text{x}}$± s, *n* = 20)

Group	7 d	14 d	28 d
Normal	0 ± 0	0 ± 0	0 ± 0
Sham	0 ± 0	0 ± 0	0 ± 0
Model	3.18 ± 0.20	3.12 ± 0.13^&^	2.48 ± 0.12^#^
NC	3.14 ± 0.11	3.10 ± 0.11^&^	2.51 ± 0.15^#^
NRSF shRNA	1.63 ± 0.07^*^	1.13 ± 0.12^*&^	0.77 ± 0.13^*#^

Note: NC, negative control; NRSF, neuron-restrictive silencer factor; d, day; ^*^P < 0.05 in comparison with the model group; ^&^*P* < 0.05 in comparison with the 7th day; ^#^*P* < 0.05 in comparison with the 14th day.

### NRSF knockdown promotes recovery of learning and memory abilities after ischemia

The results of learning and memory tests are shown in Table 2. Scores for the normal and sham groups did not differ at any of the time points. Step-down reaction periods and error times were higher, and step-down latency was lower, in the model, NC, and NRSF shRNA groups than in the normal group at all time points (all *P* < 0.05). However, these scores gradually improved in all groups as the step-down passive avoidance test progressed. Scores in the model and NC groups remained lower than those of the normal and sham groups on the 14th and 28th days (both *P* < 0.05). Scores differed on the 14th and 28th days compared to the 7th day in the NRSF shRNA group (both *P* < 0.05). Finally, scores did not differ between the model and NC groups at any of the time points, but were remarkably lower in the NRSF shRNA group than in the model and NC groups at all time points (all *P* < 0.05). These results indicate that NRSF knockdown after ischemia improved recovery of learning and memory.

**Table 2:** Comparisons of the learning and memory abilities of the rats among normal, sham, model, NC and NRSF shRNA groups (*n* = 20)

	Day	Normal	Sham	Model	NC	NRSF shRNA
Reaction time (s)	7 d	13.61 ± 8.11	12.62 ± 8.32	70.52 ± 8.24^*^	68.67 ± 8.32^*^	48.25 ± 8.90^*#^
	14 d	14.33 ± 8.06	17.52 ± 7.32	68.02 ± 7.14^*^	66.02 ± 8.14^*^	29.01 ± 7.90^*#&^
	28 d	12.48 ± 7.76	13.33 ± 7.67	31.54 ± 7.85^*&^	28.20 ± 6.78^*&^	21.19 ± 7.08^*#&^
Error times	7 d	1.36 ± 0.21	1.33 ± 0.26	4.98 ± 1.21^*^	4.87 ± 0.14^*^	3.87 ± 0.21^*#^
	14 d	1.54 ± 0.15	1.55 ± 0.31	4.94 ± 0.12^*^	4.84 ± 0.25^*^	2.94 ± 0.43^*#&^
	28 d	1.45 ± 0.19	1.45 ± 0.11	3.29 ± 0.14^*&^	3.31 ± 0.13^*&^	1.99 ± 0.14^*#&^
Latency stage (s)	7 d	269.62 ± 24.32	255.98 ± 12.44	63.46 ± 18.04^*^	54.46 ± 20.42^*^	95.43 ± 9.21^*#^
	14 d	275.91 ± 33.84	262.97 ± 27.49	78.94 ± 27.81^*^	72.65 ± 33.35^*^	193.65 ± 43.58^*#&^
	28 d	268.03 ± 34.37	259.36 ± 26.76	218.09 ± 20.51^*&^	220.21 ± 18.06^*&^	299.55 ± 19.09^*#&^
Error times	7 d	0.83 ± 0.19	0.89 ± 0.21	4.25 ± 0.16^*^	4.27 ± 0.08^*^	2.22 ± 0.13^*#^
	14 d	0.80 ± 0.15	0.76 ± 0.13	4.16 ± 0.15^*^	4.19 ± 0.13^*^	1.46 ± 0.12^*#&^
	28 d	0.78 ± 0.11	0.79 ± 0.15	1.95 ± 0.43^*&^	1.85 ± 0.69^*&^	1.04 ± 0.10^*#&^

Note: NC, negative control; NRSF, neuron-restrictive silencer factor; d, day; ^*^P < 0.05 in comparison with the normal group; ^#^*P* < 0.05 in comparison with the model group; ^&^*P* < 0.05 in comparison with previous time points.

### NRSF knockdown promotes cell proliferation and inhibits apoptosis after ischemia

BrdU immunohistochemistry (Figure 3A and 3B) revealed the presence of a small number of BrdU-positive cells in brain tissues from normal and sham group rats. After cerebral ischemia, BrdU-positive cells were also observed in the ipsilateral hippocampal dentate gyrus granule cell layer and the ependyma substratum. Many more BrdU-positive cells were present in the model, NC, and NRSF shRNA groups than in the normal group. In addition, BrdU-positive cells numbers were higher in the NRSF shRNA group than in the model group (all *P* < 0.05), but did not differ between the NC and model groups (*P* > 0.05). The results of TUNEL staining are shown in Figure 3C. Although some sporadically-distributed green fluorescence-positive apoptotic cells were present in the normal and sham groups, many more apoptotic cells, especially neurons surrounding the infarction, were present in the other three groups (Figure 3D). Apoptotic cell rates did not differ between the normal and sham groups, but were obviously higher in the other three groups than in the normal group (all *P* < 0.05). Apoptotic cell rates did not differ between in the NC and model groups, but were lower in the NRSF shRNA group than in the model group (*P* < 0.05). These results indicate that NRSF knockdown promoted proliferation and inhibited apoptosis in endogenous hippocampal nerve cells after cerebral ischemia.

**Figure 3:** BrdU-positive cell morphology (**A**), BrdU-positive cell rates (**B**), numbers of apoptotic nerve cells (**C**), and histogram of apoptosis rate (**D**) for brain tissues from each group. ^*^P < 0.05 compared to the normal group; ^#^*P* < 0.05 compared to the model group; NC, negative control; NRSF, neuron-restrictive silencer factor.

### NRSF knockdown decreases expression of apoptosis-related proteins

Western blots (Figure 4) demonstrated that Bcl-2 and Bax expression did not differ between the normal and sham groups, but were higher in the model, NC, and NRSF shRNA groups than in the normal group (all *P* < 0.05). Compared to the model group, Bcl-2 and Bax expression did not differ in the NC group, but were lower in the NRSF shRNA group (both *P* < 0.05). This indicates that apoptosis was inhibited in the NRSF shRNA group.

**Figure 4:** Expression of apoptosis-related proteins in brain tissues (**A**) and a histogram showing apoptosis-related protein expression in each group (**B**) based on Western blots. ^*^P < 0.05 compared to the normal group; ^#^*P* < 0.05 compared to the model group; NC, negative control; NRSF, neuron-restrictive silencer factor.

### NRSF knockdown upregulates MOR and DOR expression after ischemia

qRT-PCR and Western blots (Figure 5) indicated that NRSF, MOD, and DOR mRNA and protein expression did not differ between the normal and sham groups. In contrast, NRSF expression was higher and MOD and DOR expression were lower in the model group than in the normal group (all *P* > 0.05). NRSF, MOD, and DOR mRNA and protein expression did not differ between the NC and model groups. Although NRSF expression was lower and MOR and DOR expression were higher in the NRSF shRNA group than in the model group (all *P* < 0.05), no differences in expression were observed between the NRSF shRNA and normal groups. These results indicate that NRSF knockdown may affect nerve regeneration after cerebral ischemia by promoting the expression of MOR/DOR.

**Figure 5:** Histogram of NRSF and μ- and δ-opioid receptor mRNA expression (**A**), Western blot images of MOR, DOR, and NRSF expression (**B**), and histogram of NRSF, MOR, and DOR protein expression (**C**) for brain tissues from each group. ^*^P < 0.05 compared to the normal group; ^#^*P* < 0.05 compared to the model group; NRSF, neuron-restrictive silencer factor; NC, negative control; MOR, μ-opioid receptors; DOR, δ-opioid receptors.

### NRSF knockdown activates MAPK/ERK and CREB signaling pathways after ischemia

Positive staining results were observed in tissue from the cortical ischemia and hippocampal CA1 regions in the immunofluorescence assay (Figure 6A–6C). Similar levels of p-ERK and p-CREB expression were observed in the cytoplasm of normal and sham group cells (all *P* > 0.05). p-ERK expression was primarily cytoplasmic in model group cells, but nuclear expression was also observed, indicating that some nuclear translocation occurred. In contrast, p-CREB expression was primarily nuclear in model group cells. Both p-ERK and p-CREB expression were higher in the model group than in the normal group (*P* < 0.01). Although nuclear p-ERK expression was observed in cortical pyramidal neurons and the internal granular layer in the NRSF shRNA group, this expression was primarily cytoplasmic. Again, p-CREB expression was primarily nuclear in NRSF shRNA group cells. In addition, both p-ERK and p-CREB expression were higher in the NRSF shRNA group than in the model group (both *P* < 0.05). p-ERK and p-CREB expression did not differ between the NC and model groups. Western blots demonstrated that t-ERK, p-ERK, t-CREB, and p-CREB protein levels did not differ between the normal and sham groups and that t-ERK and t-CREB protein levels were similar in all of the groups (all *P* > 0.05, Figure 6D, 6E). However, p-ERK and p-CREB protein levels were higher in the model and NRSF shRNA groups than in the normal group (all *P* < 0.05). None of the protein levels examined differed between the NC and model groups. These results indicate that NRSF knockdown promoted ERK phosphorylation, which inhibited cell apoptosis and infarct development by regulating the downstream target CREB (See the Supplementary Materials).

**Figure 6:** p-ERK and p-CREB immunofluorescence in cortical ischemia and hippocampal CA1 regions (**A**), comparison of p-ERK and p-CREB expression intensity (**B**, **C**), Western blot images of t-ERK, p-ERK, t-CREB, and p-CREB proteins (**D**), and histogram of t-ERK, p-ERK, t-CREB, and p-CREB protein expression (**E**) in each. ^*^P < 0.05 compared to the normal group; ^#^*P* < 0.05 compared to the model group; NC, negative control; NRSF, neuron-restrictive silencer factor; ERK, extracellular signal-regulated kinase; CREB, response element binding protein.

### NRSF knockdown increases MAPK/ERK and CREB activation in rat NSCs after ischemia

Western blots showed that t-ERK, p-ERK, t-CREB, and p-CREB protein levels did not differ between the normal and sham groups and that t-ERK and t-CREB protein levels were similar among all groups (all *P* > 0.05, Figure 7A and 7B). However, p-ERK and p-CREB protein levels were higher in the model group than in the normal group (all *P* > 0.05). In contrast, all protein levels examined were similar in the NC and model groups (all *P* > 0.05). Finally, p-ERK and p-CREB protein levels were higher in the NRSF shRNA group than in all other groups (all *P* < 0.05).

**Figure 7:** Western blot images of t-ERK, p-ERK, t-CREB, and p-CREB proteins (**A**) and histogram of t-ERK, p-ERK, t-CREB, and p-CREB protein expression (**B**) in each group. ^*^P < 0.05 compared to the normal group; ^#^*P* < 0.05 compared to the model group; NC, negative control; NRSF, neuron-restrictive silencer factor; ERK, extracellular signal-regulated kinase; CREB, response element binding protein.

### NRSF binds directly to the μ-opioid receptor gene promoter

A chromatin immunoprecipitation (ChIP) assay was used to detect the binding of target genes to specific DNA fragments. The results showed that NRSF bound specifically to the μ opioid receptor gene promoter in rat NSCs (Figure 8).

**Figure 8:** NRSF binds to MOR/DOR promoter genes Paraformaldehyde cross-linking was performed after chromatin from rat brain neural stem cells was cut into fragments of BP 200~2000 using sonication (**A**); Chromatin and ChIP antibodies were separated by shear after immunoprecipitation, and purified DNA introns were amplified using PCR (**B**). NRSF, neuron-restrictive silencer factor; MOR/DOR, μ- and δ-opioid receptors; ChIP, chromatin immunoprecipitation assay.

### Detection of packaging and lentiviral vector titer

As expected, all 3 positive clones selected for qRT-PCR review had positive bands (343 bp) (Supplementary Figure 1A). After being exposed to the virus, cytopathic effects (CPE) were observed in 293 T cells under an inverted microscope; cells and nuclei became extended and round and cell attachment decreased (Supplementary Figure 1B). The titer was 2 × 10^8^ TU/L.

## DISCUSSION

Cerebral ischemia is the major cause of swelling in the brain and breakdown of the blood-brain barrier [18]. Extensive research indicates that ischemic stroke triggers a series of biochemical events that lead to necrotic and apoptotic neuronal death in ischemic regions [19]. Illumination of the molecular mechanisms behind cell apoptosis might provide new insights into cerebral ischemia and improve the efficacy of clinical therapeutic strategies.

In this study, neurological function scores and step-down reaction periods were lower, and step-down latencies were higher, in NRSF shRNA group rats than in model and NC group rats. This indicated that NRSF knockdown accelerated recovery of neurological function and improved learning and memory after ischemia. Several studies have examined the relationship between NRSF and brain ischemia. Calderone *et al*. reported that global ischemia triggered NRSF mRNA and protein expression [20]. A recent study demonstrated that NRSF was one of the protein complexes that modulated Na^+^-Ca2^+^ exchanger 1 expression during brain ischemia and ischemic preconditioning [21]. Interestingly, Formisano *et al*. found that ischemia promoted association of NRSF with the MOR-1 promoter in vulnerable CA1 neurons [22]. NRSF is repressor element-1 silencing transcription factor and plays a vital role in neurogenesis and embryonic development [23]. NRSF binds to a 21-nt DNA sequence named NRSF or repressor element-1 (RE1). In the human and mouse genomes, NRSF sequences are present in many genes and are especially abundant in genes that encode nervous system constituents, such as neurotransmitter receptors, ion channels, and synaptic transmission factors [24]. During neurogenesis, downregulation of NRSF expression enhanced the transcription of its target genes, which were important for neuronal differentiation [25]. NRSF downregulation also altered the expression of NRSF-regulated hippocampal genes, such as receptors, calcium-related molecules, ion channels, and other transcription factors, that control neuronal function and plasticity [26]. Because the hippocampus is critical for spatial memory and learning [27], inhibition of NRSF might promote hippocampal gene expression and improve learning and memory abilities after cerebral ischemia. Gupta *et al*. demonstrated that downregulation of NRSF could increase numbers of mature neurons [28]; this may be important because neurons at different maturation stages make distinct contributions to processes of learning and memory [29].

Additionally, apoptosis rates and Bcl-2 and Bax expression were lower, while BrdU-positive cell numbers were higher, in rats in the NRSF shRNA group compared to the other groups. This indicated that NRSF knockdown promoted proliferation and inhibited apoptosis in endogenous neurons. NRSF represses neuronal promoters and triggers apoptosis by activating caspase cascades [30]. NRSF also functions as a repressor in neuronal cells by binding to the NRSF of the MOR gene in a sequence-specific manner [31]. The interaction of NRSF with 3 binding sites and NRSF2 is also responsible for N-methyl-D-aspartic acid receptor 2B (NR2B) gene repression [32]. NR2B activation is both important during the priming stage for prevention and a target for the effective treatment of ischemic cell damage [33]. It is therefore possible that NRSF knockdown disinhibited NR2B expression, resulting in decreased apoptosis rates. In line with these findings, Dave *et al*. demonstrated that an NR2B receptor antagonist had anti-apoptotic effects [34]. The Bcl-2 family of proteins is essential in regulating apoptosis and controling cellular fate in response to numerous stress signals and developmental cues [35], and Bax is a pro-apoptotic protein in the Bcl-2 family [36]. It is possible that NRSF knockdown reduces apoptosis by decreasing Bax expression. The Bcl-2 is an anti-apoptotic protein also protects cells from programmed death [37]. The cause of the reductions in Bcl-2 expression that accompanied reductions in apoptosis rates in this study remains unclear and should be investigated in future studies. The BrdU labeling assay is widely used to evaluate cell proliferation [38], and cells stained with BrdU are either new or in the process of dividing [39]. Our results indicate that NRSF knockdown increases numbers of new-born cells, which is indicative of lower apoptosis rates.

Increased MOR/DOR expression and decreased NRSF expression were observed in the NRSF shRNA group. MOR is a G protein-coupled receptor which is activated by opioids and endogenous opioid peptides. Clinical and pharmacological studies demonstrate that MOR is the main site of action for many major clinical analgesics, such as morphine [40]. The synergistic interaction between NRSF and Sp3 inhibits MOR gene transcription [41]. Here, NRSF knockdown resulted in a disinhibition of MOR gene transcription. The δ-opioid receptor (DOR) is expressed in limbic structures and cortical regions, such as the amygdala, hippocampus, hypothalamus, and basal ganglia, in the human central nervous system [42]. Analgesia induced by DOR ligands is mediated by the MOR [43], and MOR expression is positively correlated with DOR expression. Furthermore, MOR/DOR agonists stimulated the proliferation of isolated rat adult hippocampal progenitor neurons [44]. These findings are in accordance with the observation that NRSF knockdown promoted cell proliferation in this study. We therefore believe that MOR/DOR expression was an important regulator of cell proliferation here. However, few studies have examined direct links between NRSF and DOR expression and activity, and further investigation is needed to confirm our findings.

In this study, p-ERK and p-CREB expression were also elevated in the NRSF shRNA group. This indicated that NRSF knockdown promoted ERK phosphorylation, regulated its downstream target CREB, and inhibited cell apoptosis. Ethanol-induced potentiation of NRSF binding activity can inhibit ERK phosphorylation without affecting total ERK expression [45], which is consistent with the present results. NRSF knockdown also upregulates MAPK/ERK signaling and promotes the expression of mesendodermal differentiation markers [46]. ERK in turn phosphorylates CREB by activating ribosomal S6 kinase and mitogen and stress activated protein kinase [47]. Once it is activated by phosphorylation [48], CREB regulates the anti-apoptotic gene and myeloid cell leukemia sequence 1 (Mcl-1). Furthermore, inhibition of CREB triggers apoptotic nerve cell death [49]. This may explain, at least in part, the decrease in apoptosis that accompanied increased p-CREB expression in the NRSF shRNA group in this study.

In conclusion, NRSF knockdown accelerates recovery of neurological function and learning and memory processes, promotes proliferation, and surpresses apoptosis in endogenous neurons after ischemia. These results suggest that NRSF may be a promising target in the treatment of cerebral ischemia. Although several previous studies indicate that MOR-DOR interactions modulate ligand binding, receptor signaling, and trafficking properties, and the ChIP assay performed here confirmed an interaction between MOR and NRSF. Additional ChIP assays are needed to examine whether NRSF binds to DORs; such studies would further elucidate the mechanistic link between NRSF and MOR/DOR and their impact on proliferation and apoptosis in endogenous NSCs.

## MATERIALS AND METHODS

### Ethics statement

All experiments adhered strictly to basic animal welfare principles, the “3R” (replacement, reduction and refinement) principles, and the ethical requirements of animal experiments.

### Establishment and identification of the NRSF shRNA lentiviral vector

NRSF shRNA (GAAGAACAGTTTGTGCATC) and scramble shRNA (GACAGAGTAATTCCGAGTT) were designed based on the NRSF sequence in the GeneBank database and synthesized by Shanghai Sangon Biological Engineering Technology & Services Co., Ltd. (Shanghai, China). HpaI and XhoI were used to digest the pFU-GW-RNAi plasmid (GeneChem Co. Ltd, Shanghai, China) and the product of this digestion was connected to the shRNA using ligase T4 DNA to obtain NRSF shRNA and scramble shRNA recombinant plasmids. Recombinant plasmids were then amplified using polymerase chain reaction (PCR) and collected for sequence detection. The primer sequences were 5′-GCCCCGGTTAATGCATAT-3′ (forward) and 5′-GAGGCCAGATCTTGGGTG-3′ (reverse) (Supplementary Figure 1). After being incubated for 20 mins, a mixture of recombinant plasmids and Lipofectamine 2000 solution was transferred into cultures of 293T cells. Eight hours later, the medium was removed, 10% fetal bovine serum (FBS) was added, and culture continued for another 48 hrs. The 293T cell supernatant was collected, filtered (0.45 μm), and then centrifuged at 25000 r/min for 20 mins at 4°C. Ice-cold phosphate buffer solution (PBS) was used to precipitate transfected cells. After being lysed and stored at 4°C overnight, the cells were separated into tubes (10 μL each) and stored at −80°C. 293T cells were cultured for 24 hrs in transfection solution diluted with serum-free medium, 100 μL of complete medium was added, and the cytopathic effect (CPE) was measured 10 days later. Wells with CPEs were counted and the CPE-positive rate was calculated for each group. The virus titer was calculated using the Karber method: titer (T) = 10^1 + d (s-0.5)^, where d = log_10_(dilution) and s = the sum of positive rate.

### Cerebral blood flow (CBF) measurement

A total of 100 male Sprague-Dawley (SD) rats (weighing about 230 g) were purchased from the experimental animal center at the Chinese Academy of Sciences (Shanghai, China); animals were fed a normal diet and maintained under a normal light cycle. The rats were randomly distributed among the following 5 groups of 20 rats each: normal, sham, model, negative control (NC), and NRSF shRNA interference (NRSF shRNA). The rats were fasted for 12 hrs and their right middle cerebral arteries were then blocked using the suture method [50] to produce ischemia. After anesthesia was administered (chloral hydrate 350 mg/kg), a midline incision was made on the neck. The bottom of the right internal and external carotid artery was exposed and a 4–0 nylon surgical suture (Davis & Geck, Wayne, NJ, USA) was inserted at the entrance of cerebral artery. After 1 hr of ischemia, the nylon suture was removed to allow reperfusion. A laser Doppler flow meter (PeriFlux 5000, Perimed, Stockholm, Sweden) was used to measure regional CBF in the cortex. The laser Doppler flow meter was fixed in the brain 2 mm from midline and 1 mm from the coronal suture. An initial decline in CBF followed by stabilization indicated that the ischemia model was successful. During the experiment, rat body temperature was kept at 37°C using electric light and a thermal insulation blanket. Rats in the normal group received injections of artificial cerebral spinal fluid into the lateral ventricles instead of ischemia. Rats in the sham group received injections of artificial cerebral spinal fluid into the lateral ventricles and underwent vascular separation without ischemia treatment; no nylon sutures were inserted into the skull. Rats in the model group underwent ischemia and received artificial cerebrospinal fluid injections into the lateral ventricles. Rats in the NC group underwent ischemia and received injections of cerebrospinal fluid with the scramble shRNA sequence into the lateral ventricles. Rats in the NRSF shRNA group underwent ischemia and received injections of the cerebrospinal fluid with the NRSF shRNA sequence cerebrospinal fluid was injected into the lateral ventricles.

### Neurological function scoring

Neurological function scoring was performed according to the Zealonga method [50]. An experimenter without knowledge of the group assignments assessed neurological deficits on the 7th, 14th, and 28th days after ischemia and reperfusion. The severity of injury increases as the score increases. The scores were as follows: 0, normal, no neurological sign; score 1, cannot completely stretch contralateral forelimbs; score 2, contralateral circling when walking; score 3, contralateral fall over when walking; score 4, cannot walk, reduced consciousness.

### Step-down passive avoidance test

On the 7th, 14th, and 28th days after ischemia and reperfusion, rats were placed in the step-down apparatus (Ji Xing Instrument Technology Development Co., Ltd, Shijiazhuang, Hebei, China). They were habituated to the environment for 3 mins and were then subjected to electric shock from an alternating current. The amount of time a rat took to jump back to the safety board was defined as the step-down reaction period. The number of times a rat received an electric shock within 5 mins was defined as the number of errors. Step-down reaction period and number of errors were used to evaluate learning ability. 24 hrs later, the experiment was repeated. The rats received an electric shock as soon as they were placed in the chamber. The amount of time a rat took to jump from the copper bar to the board was defined as the step-down latency; trials were ended after 5 minutes if the rat had not jumped. The number of times a rats received electric shocks was defined as the number of errors. Step-down latency and the number of errors were used to evaluate the memory ability of the rats.

### Sample collection

The rats were sacrificed on the 28th day after ischemia and reperfusion. Rats were given three intraperitoneal injections of bromodeoxyuridine (BrdU, 50 mg/kg, Sigma-Aldrich Chemical Company, St Louis MO, USA) in 4 hr intervals 12 hrs before sacrifice. After the final injection, the rats were deeply anesthetized by an intraperitoneal injection of sodium pentobarbital (50 mg/kg). The rats were then decapitated and the cerebral cortex and nipped leptomeningeal and vascular tissues were removed under an anatomic microscope. The brain tissues were cut into 1 mm3 pieces, digested with 125% trypsin and 0.01% EDTA for 10 min, and transferred to FBS to make cell suspensions for further use. Subsequently, a portion of the tissue was removed and stored at −80°C for use in quantitative real-time polymerase chain reaction (qRT-PCR) and western blotting. The remaining tissue was fixed with 4% triformol for 24 hrs and sliced into coronal sections at the level of the hippocampus infarct area. Next, the sections were dehydrated using alcohol and immersed in a paraffin box for full fixation. The embedding device was then placed on an ice block to completely cool the brain tissues. Finally, the frozen brain tissues were sliced into coronal sections (4 μm thick) and stored at 4°C for immunohistochemistry and Terminal-deoxynucleotidyl Transferase Mediated Nick End Labeling (TUNEL) staining.

### Immunohistochemistry

The frozen sections were dewaxed and dehydrated with alcohol, and 3% hydrogen peroxide was then used to quench endogenous peroxidase. The sections were then microwaved for 30 mins in a 0.01 M citrate buffer solution (pH 6.0) for antigen retrieval. After cooling to room temperature, the sections were rinsed with PBS. Next, the rabbit anti-mouse BrdU monoclonal antibody (1:50, Labvision Corp., Fremont, CA, USA) was added and incubated at 37°C for 1 hr. Biotinylated goat anti-rabbit second antibody was then added and incubated at 37°C for 30 mins. Sections were then incubated with diaminobenzidine (DBA) for 1~2 mins, rinsed again 3 times with PBS (2 mins/rinse), re-dyed for 1 min with hematoxylin, dehydrated, mounted, and sealed. Known positive sections served as positive controls and the primary antibody was replaced with PBS for the negative control. The cells with yellowish-brown granules in the cytoplasm or nuclei were considered positive cells. Positive cells were counted in five randomly-selected fields under high magnification (× 400); positive cell rate = the number of positive cells/the total number of cells × 100%. Immunohistochemistry quantification was performed independently by two double-blind experimenters.

### TUNEL assay

Apoptotic cells were quantified in rat brain tissues according to the instructions of the DeadEnd^TM^ fluorescence labeling TUNEL detection kit (Promega Corp., Madison, WI, USA). Cells were rinsed 3 times with PBS for 4 mins each. After excess liquid evaporated, 100 μL of equilibration buffer was added and incubated for 10 mins. Excess liquid was then removed and 100 μL of TdT enzyme was slowly added to the mixture, followed by incubation for 60 mins at 37°C and a PBS rinse. The stop solution was then added and incubated for 10 mins followed by a PBS rinse. The cells were pre-stained with 4,6-2 amidine base-2-phenyl indole (DAPI, 10 mg/mL) for 5 mins at room temperature and rinsed with PBS. Cells were then examined under a laser scanning confocal microscope (Nikon Instech, Co., Ltd, Karagawa, Japan); nuclei were stained blue with DAPI and apoptotic cells were stained green. Apoptotic cells were counted in five randomly-selected fields under high magnification (× 400) using the ImageProPlus image analysis and processing system (Motic Med 6.0 system, USA); apoptotic cell rate = the number of green apoptotic cells/the total number of blue cells × 100%.

### Immunofluorescence

Brain sections were heated at 65°C for 30 mins, dewaxed, dehydrated, and rinsed with PBS. Sections were then immersed in a sodium citrate buffer solution (0.01 mol/L), boiled for 12 mins, and re-rinsed with PBS after cooling. Sections were then incubated with 500 μL of 3% Tritonx-100 for 30 mins to enhance permeability. The sections were then rinsed with PBS and blocked with ready-to-use goat serum for 40 mins. P-extracellular signal-regulated kinase (ERK, 1: 200) and p-responsive element-binding protein (CREB) rabbit polyclonal antibodies were added and incubated overnight at 4°C. Sections were then rinsed with PBS and incubated in a wet box with 100 μL of goat anti-rabbit secondary antibody labeled with tetraethyl rhodamine isothiocyanate (TRITC, 1: 50) for 1 hr at 37°C in the dark, followed by another PBS rinse. Sections were then dried with filter paper and sealed with mounting medium containing DAPI. The sections were observed under a laser scanning confocal microscope (Nikon Corporation, Japan). DAPI-labeled nuclei were blue, while cells labeled by the secondary antibody were red. In each group, five randomly-selected high-magnification fields (× 400) were analyzed using the ImageProPlus image processing and analysis system (Motic Med 6.0 system, USA); DAPI and immunohistochemical staining were overlapped and the background was corrected based on which positive fluorescence intensity was being analyzed.

### Quantitative real-time polymerase chain reaction (qRT-PCR)

Total RNA was extracted from rat NSCs according to the instructions provided with the TRIZOL kit (Invitrogen, Inc., Carlsbad, CA, USA). An ultraviolet spectrophotometer (Nanodrop Technologies, Wilmington, DE, USA) was used to measure the absorbance at 260 nm and 280 nm, and total RNA quality was examined. The PrimeScript@RT reagent Kit (PerfectRealTime) (Takara Biotechnology Ltd., Dalian, China) was used to reverse-transcribe total RNA into cDNA, which was then used for PCR amplification. The following primer sequences were used: NRSF: 5′-ATTGAAGTTGGCTTAGTG-3′ (forward) and 5′-TATGGGTAGATTCGTTGA-3′ (reverse); μ-opioid receptor: 5′-GAATCGTCCGGTACACTAAGC-3′ (forward) and 5′-GTCACTGCCATGACCATGATG-3′ (reverse); δ-opioid receptor: 5′-GAATCGTCCGGTACACTAAGC-3′ (forward) and 5′-GTCACTGCCATGACCATGATG-3′ (reverse); and β-actin: 5′-CACCCGCGAGTACAACCTTC-3′ (forward) and 5′-CCCATACCCACCATCACACC-3′ (reverse). The PCR amplification reaction system (50 μL) included 5 μL 10 × PCR buffer solution, 1 μL dNTPs, 6 μL MgCl_2_, 1 μL forward and reverse primers, 0.5 μL TaqDNA polymerase, 2.5 μL reverse primers, and 50 μL EDPC water. The reaction conditions consisted of 40 cycles of pre-denaturation at 95°C for 5 mins, denaturation at 90°C for 30 s, annealing at 60°C for 40 s, and extension at 72°C for 40 s. All data were analyzed using the 2^-ΔΔCt^ method; ΔΔCT = ΔCt _experimental group_ – ΔCt _control group_, and ΔCt = Ct _target gene_ – Ct _β-actin_ [51].

### Western blotting

Protein lysate (Shanghai Beyotime Biotechnology Co., Shanghai, China) was added to the NSCs and frozen brain tissues to extract total protein. The Bradford method (Thermo Fisher Scientific Inc., Waltham, MA, USA) was used to assess protein quality. Total protein (50 μg) was then used for 12% SDS-PAGE (sodium dodecyl sulfate polyacrylamide gel electrophoresis) electrophoresis and transferred onto PVDF membranes (Millipore, Billerica, MA, USA). After blocking with 5% skim milk at 37°C for 1 hr, the membranes were incubated with rabbit anti-mouse NRSF (ab21635,1: 500), MOR (ab1009,1: 700), DOR (ab83775, 1: 1,000), Bcl-2 (ab32124,1: 1,000), Bax (ab32053, 1: 1,000), and β-actin (ab8227, 1: 1,000) monoclonal antibodies (Abcam, Inc., Cambridge, MA, USA) overnight at 4°C. Membranes were then rinsed with tris-buffered saline Tween-20 (TBST) 3 times for 5 min and horse radish peroxidase (HRP) labelled goat anti-rabbit second antibody (ab20272, 1: 4000; Abcam, Inc., Cambridge, MA, USA) was added. The membrane was incubated for 2 hrs at room temperature and then rinsed. Relative protein expression was quantified by comparing the gray value of the target band to the internal reference band.

### ChIP assay

Specific binding between MOR and NRSF was detected according to the instructions of the ChIP Assay Kit (Qiagen company, Hilden, Germany). Cells were cross linked by adding 1% formaldehyde and cooled in 0.125 M glycine solution. DNA was then immunoprecipitated using rabbit anti-rat antibody or control antibody and then used for qRT-PCR assay. The primer sequences for MOR were 5-CTGTGAGAGGAAGAGGCTG-3′ (forward) and 5-AAGTTGAGCCAGGAGCCAGGT-3′ (reverse); the product was 118bp in length.

### Statistical analysis

SPSS 20.0 software (SPSS Inc. Chicago, IL, USA) was used for data analysis. Continuous data are expressed as means ± standard deviation (SD) and *t* tests were used for comparisons between groups. Enumeration data are expressed as percentages or ratios and were compared using the χ^2^-test. Comparisons among multiple groups were performed using analysis of variance (ANOVA) and homogeneity of variance was examined. When significant differences were identified by ANOVAs, the *q*-test was used for further comparisons between two groups. When heterogeneous variance was detected, the nonparametric rank test was used for analysis with α = 0.05. *P* < 0.05 was considered statistically significant.

## SUPPLEMENTARY MATERIALS FIGURE



## References

[1] Zhang J, Li X, Chai S, Wang X (2015). Neuroprotective effect of lentivirus mediated VEGF on rat model with cerebral ischemic injury. Int J Clin Exp Med.

[2] Wang YS, Li YX, Zhao P, Wang HB, Zhou R, Hao YJ, Wang J, Wang SJ, Du J, Ma L, Sun T, Yu JQ (2015). Anti-inflammation Effects of Oxysophoridine on Cerebral Ischemia-Reperfusion Injury in Mice. Inflammation.

[3] Guo Y, Xu X, Li Q, Li Z, Du F (2010). Anti-inflammation effects of picroside 2 in cerebral ischemic injury rats. Behav Brain Funct.

[4] Nardi K, Engelter S, Strbian D, Sarikaya H, Arnold M, Casoni F, Ford GA, Cordonnier C, Lyrer P, Bordet R, Soinne L, Gensicke H, Duriez P (2012). Lipid profiles and outcome in patients treated by intravenous thrombolysis for cerebral ischemia. Neurology.

[5] Zhao J, Yu S, Zheng W, Feng G, Luo G, Wang L, Zhao Y (2010). Curcumin improves outcomes and attenuates focal cerebral ischemic injury via antiapoptotic mechanisms in rats. Neurochem Res.

[6] Pei H, Su X, Zhao L, Li H, Guo Y, Zhang M, Xin H (2012). Primary study for the therapeutic dose and time window of picroside II in treating cerebral ischemic injury in rats. Int J Mol Sci.

[7] Shi H, Sun BL, Zhang J, Lu S, Zhang P, Wang H, Yu Q, Stetler RA, Vosler PS, Chen J, Gao Y (2013). miR-15b suppression of Bcl-2 contributes to cerebral ischemic injury and is reversed by sevoflurane preconditioning. CNS Neurol Disord Drug Targets.

[8] Kreisler A, Strissel PL, Strick R, Neumann SB, Schumacher U, Becker CM (2010). Regulation of the NRSF/REST gene by methylation and CREB affects the cellular phenotype of small-cell lung cancer. Oncogene.

[9] Atouf F, Czernichow P, Scharfmann R (1997). Expression of neuronal traits in pancreatic beta cells. Implication of neuron-restrictive silencing factor/repressor element silencing transcription factor, a neuron-restrictive silencer. J Biol Chem.

[10] Yang YJ, Baltus AE, Mathew RS, Murphy EA, Evrony GD, Gonzalez DM, Wang EP, Marshall-Walker CA, Barry BJ, Murn J, Tatarakis A, Mahajan MA, Samuels HH (2012). Microcephaly gene links trithorax and REST/NRSF to control neural stem cell proliferation and differentiation. Cell.

[11] Kieffer BL (1995). Recent advances in molecular recognition and signal transduction of active peptides: receptors for opioid peptides. Cell Mol Neurobiol.

[12] Fujita W, Gomes I, Devi LA (2015). Heteromers of mu-delta opioid receptors: new pharmacology and novel therapeutic possibilities. Br J Pharmacol.

[13] Chen YL, Law PY, Loh HH (2008). The other side of the opioid story: modulation of cell growth and survival signaling. Curr Med Chem.

[14] Choi IY, Ju C, Anthony Jalin AM, Lee DI, Prather PL, Kim WK (2013). Activation of cannabinoid CB2 receptor-mediated AMPK/CREB pathway reduces cerebral ischemic injury. Am J Pathol.

[15] Xiong LZ, Yang J, Wang Q, Lu ZH (2007). Involvement of delta-and mu-opioid receptors in the delayed cerebral ischemic tolerance induced by repeated electroacupuncture preconditioning in rats. Chin Med J (Engl).

[16] Husain S, Potter DE, Crosson CE (2009). Opioid receptor-activation: retina protected from ischemic injury. Invest Ophthalmol Vis Sci.

[17] Song KY, Choi HS, Law PY, Wei LN, Loh HH (2012). Post-transcriptional regulation of mu-opioid receptor: role of the RNA-binding proteins heterogeneous nuclear ribonucleoprotein H1 and F. Cell Mol Life Sci.

[18] Rosenberg GA, Yang Y (2007). Vasogenic edema due to tight junction disruption by matrix metalloproteinases in cerebral ischemia. Neurosurg Focus.

[19] Yin KJ, Deng Z, Huang H, Hamblin M, Xie C, Zhang J, Chen YE (2010). miR-497 regulates neuronal death in mouse brain after transient focal cerebral ischemia. Neurobiol Dis.

[20] Calderone A, Jover T, Noh KM, Tanaka H, Yokota H, Lin Y, Grooms SY, Regis R, Bennett MV, Zukin RS (2003). Ischemic insults derepress the gene silencer REST in neurons destined to die. J Neurosci.

[21] Formisano L, Guida N, Valsecchi V, Cantile M, Cuomo O, Vinciguerra A, Laudati G, Pignataro G, Sirabella R, Di Renzo G, Annunziato L (2015). Sp3/REST/HDAC1/HDAC2 Complex Represses and Sp1/HIF-1/p300 Complex Activates ncx1 Gene Transcription, in Brain Ischemia and in Ischemic Brain Preconditioning, by Epigenetic Mechanism. J Neurosci.

[22] Formisano L, Noh KM, Miyawaki T, Mashiko T, Bennett MV, Zukin RS (2007). Ischemic insults promote epigenetic reprogramming of mu opioid receptor expression in hippocampal neurons. Proc Natl Acad Sci USA.

[23] Hu XL, Cheng X, Cai L, Tan GH, Xu L, Feng XY, Lu TJ, Xiong H, Fei J, Xiong ZQ (2011). Conditional deletion of NRSF in forebrain neurons accelerates epileptogenesis in the kindling model. Cereb Cortex.

[24] Bruce AW, Donaldson IJ, Wood IC, Yerbury SA, Sadowski MI, Chapman M, Gottgens B, Buckley NJ (2004). Genome-wide analysis of repressor element 1 silencing transcription factor/neuron-restrictive silencing factor (REST/NRSF) target genes. Proc Natl Acad Sci USA.

[25] Ballas N, Grunseich C, Lu DD, Speh JC, Mandel G (2005). REST and its corepressors mediate plasticity of neuronal gene chromatin throughout neurogenesis. Cell.

[26] McClelland S, Brennan GP, Dube C, Rajpara S, Iyer S, Richichi C, Bernard C, Baram TZ (2014). The transcription factor NRSF contributes to epileptogenesis by selective repression of a subset of target genes. Elife.

[27] Ohshima T, Ogura H, Tomizawa K, Hayashi K, Suzuki H, Saito T, Kamei H, Nishi A, Bibb JA, Hisanaga S, Matsui H, Mikoshiba K (2005). Impairment of hippocampal long-term depression and defective spatial learning and memory in p35 mice. J Neurochem.

[28] Gupta SK, Gressens P, Mani S (2009). NRSF downregulation induces neuronal differentiation in mouse embryonic stem cells. Differentiation.

[29] Deng W, Aimone JB, Gage FH (2010). New neurons and new memories: how does adult hippocampal neurogenesis affect learning and memory?. Nat Rev Neurosci.

[30] Lawinger P, Venugopal R, Guo ZS, Immaneni A, Sengupta D, Lu W, Rastelli L, Marin Dias Carneiro A, Levin V, Fuller GN, Echelard Y, Majumder S (2000). The neuronal repressor REST/NRSF is an essential regulator in medulloblastoma cells. Nat Med.

[31] Kim CS, Hwang CK, Choi HS, Song KY, Law PY, Wei LN, Loh HH (2004). Neuron-restrictive silencer factor (NRSF) functions as a repressor in neuronal cells to regulate the mu opioid receptor gene. J Biol Chem.

[32] Pignataro L, Varodayan FP, Tannenholz LE, Harrison NL (2009). The regulation of neuronal gene expression by alcohol. Pharmacol Ther.

[33] Liu Z, Zhao W, Xu T, Pei D, Peng Y (2010). Alterations of NMDA receptor subunits NR1, NR2A and NR2B mRNA expression and their relationship to apoptosis following transient forebrain ischemia. Brain Res.

[34] Dave JR, Williams AJ, Moffett JR, Koenig ML, Tortella FC (2003). Studies on neuronal apoptosis in primary forebrain cultures: neuroprotective/anti-apoptotic action of NR2B NMDA antagonists. Neurotox Res.

[35] Chen L, Willis SN, Wei A, Smith BJ, Fletcher JI, Hinds MG, Colman PM, Day CL, Adams JM, Huang DC (2005). Differential targeting of prosurvival Bcl-2 proteins by their BH3-only ligands allows complementary apoptotic function. Mol Cell.

[36] Xu Q, Dou J, Wei P, Tan C, Yun X, Wu Y, Bai X, Ma X, Du Y (2008). Chitooligosaccharides induce apoptosis of human hepatocellular carcinoma cells via up-regulation of Bax. Carbohydrate Polymers.

[37] Bedikian AY, Millward M, Pehamberger H, Conry R, Gore M, Trefzer U, Pavlick AC, DeConti R, Hersh EM, Hersey P, Kirkwood JM, Haluska FG, Oblimersen Melanoma Study Group (2006). Bcl-2 antisense (oblimersen sodium) plus dacarbazine in patients with advanced melanoma: the Oblimersen Melanoma Study Group. J Clin Oncol.

[38] Ferretti E, De Smaele E, Po A, Di Marcotullio L, Tosi E, Espinola MS, Di Rocco C, Riccardi R, Giangaspero F, Farcomeni A, Nofroni I, Laneve P, Gioia U (2009). MicroRNA profiling in human medulloblastoma. Int J Cancer.

[39] Bartley J, Soltau T, Wimborne H, Kim S, Martin-Studdard A, Hess D, Hill W, Waller J, Carroll J (2005). BrdU-positive cells in the neonatal mouse hippocampus following hypoxic-ischemic brain injury. BMC Neurosci.

[40] Kim CS, Hwang CK, Song KY, Choi HS, Kim DK, Law PY, Wei LN, Loh HH (2008). Novel function of neuron-restrictive silencer factor (NRSF) for posttranscriptional regulation. Biochim Biophys Acta.

[41] Kim CS, Choi HS, Hwang CK, Song KY, Lee BK, Law PY, Wei LN, Loh HH (2006). Evidence of the neuron-restrictive silencer factor (NRSF) interaction with Sp3 and its synergic repression to the mu opioid receptor (MOR) gene. Nucleic Acids Res.

[42] Chu Sin Chung P, Kieffer BL (2013). Delta opioid receptors in brain function and diseases. Pharmacol Ther.

[43] Rozenfeld R, Abul-Husn NS, Gomez I, Devi LA (2007). An emerging role for the delta opioid receptor in the regulation of mu opioid receptor function. ScientificWorldJournal.

[44] Persson AI, Thorlin T, Bull C, Eriksson PS (2003). Opioid-induced proliferation through the MAPK pathway in cultures of adult hippocampal progenitors. Mol Cell Neurosci.

[45] Tateno M, Ukai W, Hashimoto E, Ikeda H, Saito T (2006). Implication of increased NRSF/REST binding activity in the mechanism of ethanol inhibition of neuronal differentiation. J Neural Transm (Vienna).

[46] Thakore-Shah K, Koleilat T, Jan M, John A, Pyle AD (2015). REST/NRSF Knockdown Alters Survival, Lineage Differentiation and Signaling in Human Embryonic Stem Cells. PLoS One.

[47] Kenney JW, Poole RL, Adoff MD, Logue SF, Gould TJ (2012). Learning and nicotine interact to increase CREB phosphorylation at the jnk1 promoter in the hippocampus. PLoS One.

[48] Xia Z, Storm DR (2005). The role of calmodulin as a signal integrator for synaptic plasticity. Nat Rev Neurosci.

[49] Sakamoto K, Karelina K, Obrietan K (2011). CREB: a multifaceted regulator of neuronal plasticity and protection. J Neurochem.

[50] Zhao P, Huang ZN, Chen G, Cheng JS (2000). Electro-acupuncture attenuates nitric oxide release from rat striatum after transient middle cerebral artery occlusion. Acupunct Electrother Res.

[51] Kim YK, Shin DH, Kim KB, Shin N, Park WY, Lee JH, Choi KU, Kim JY, Lee CH, Sol MY, Kim MH (2015). MUC5AC and MUC5B enhance the characterization of mucinous adenocarcinomas of the lung and predict poor prognosis. Histopathology.

